# Prediabetes predicts adverse cardiovascular outcomes after percutaneous coronary intervention: a meta-analysis

**DOI:** 10.1042/BSR20193130

**Published:** 2020-01-07

**Authors:** Yong Zhao, Min Guo, Gang Shi

**Affiliations:** 1 Department of Cardiology, Pingxiang People’s Hospital, Pingxiang 337000, China; 2 Department of Respiration, General Hospital of Pingxiang Mining Industry Group Co., Ltd., Pingxiang 337000, China

**Keywords:** coronary artery disease, major adverse cardiovascular events, meta-analysis, percutaneous coronary intervention, prediabetes

## Abstract

**Background:** Prediabetes has been related with increased risk of coronary artery disease (CAD). However, the prognostic efficacy of prediabetes for patients receiving percutaneous coronary intervention (PCI) remains undetermined. We aimed to quantitatively evaluate the influence of diabetes on the risks of major adverse cardiovascular events (MACEs) after PCI in a meta-analysis.

**Methods:** Longitudinal follow-up studies evaluating the association between prediabetes and risks of MACEs and mortality after PCI were identified by search of PubMed and Embase databases. A random-effect model was applied to pool the results. Subgroup analyses were performed to evaluate the impacts of study characteristics on the outcome.

**Results:** Twelve follow-up studies including 10,048 patients that underwent PCI were included. Compared with patients with normoglycemia at admission, those with prediabetes were had significantly higher risk MACEs during follow-up (adjusted risk ratio [RR]: 1.53, 95% confidence interval [CI]: 1.25–1.87, *P* < 0.001). Further subgroup analyses indicated that the association between prediabetes and higher risk of MACEs remained regardless of the study design, sample size, CAD subtype, PCI type, definition of diabetes, or follow-up duration. Moreover, patients with prediabetes had higher significantly risk of MACEs in studies with adjustment of coronary lesion severity (RR: 1.79, *P* < 0.001), but the association became insignificant in studies without adjustment of the coronary lesion severity (RR: 1.23, *P* = 0.09).

**Conclusions:** Prediabetes is independently associated with increased risk of MACEs after PCI as compared with those with normoglycemia, even in studies with adjustment of coronary severity.

## Introduction

Diabetes mellitus (DM) has been confirmed to confer equivalent mortality risk as coronary artery disease (CAD) in clinical practice [1–3]. Moreover, as a prevalent metabolic disease, DM is not only recognized as a major risk factor for CAD development, but also established as an independent predictor of poor prognosis in CAD patients [4]. A recent meta-analysis including 139,774 CAD patients after percutaneous coronary intervention (PCI) showed that DM is independently associated with worse short-term and long-term prognosis [5]. Recent evidence suggests that besides of patients with DM, those with prediabetes are also vulnerable to atherosclerotic cardiovascular diseases [6,7]. Prediabetes refers to the moderately impaired glycemic metabolism that does not fulfill the current diagnostic criteria of DM. Currently, prediabetes mainly includes impaired fasting glucose (IFG) and impaired glucose tolerance (IGT) [8]. Although IGT is consistently defined as a 2-h plasma glucose concentration of 7.8–11.0 mmol/l during an oral glucose tolerance test, the definitions of IFG are different according to the World Health Organization (WHO) criteria (fasting plasma glucose [FPG]: 6.1–6.9 mmol/l) and the 2003 American Diabetes Association (ADA) guideline criteria (FPG: 5.6–6.9 mmol/l) [8]. Moreover, the glycosylated hemoglobin (HbA1c) of 5.7–6.4% and 6.0–6.4% has also been considered as definitions for prediabetes by ADA and National Institute for Health and Care Excellence (NICE), respectively [9,10]. Despite of the varying definitions, people with prediabetes confirmed to have significantly increased risks of CAD, stroke, and all-cause mortality as compared those with normoglycemia [11]. However, studies reporting the association between prediabetes and clinical outcomes of CAD patients after PCI showed inconsistent results [12–23]. Although results of some studies supported that prediabetes was a potential predictor of poor prognosis in patients after PCI [12–14,18,21], others did not find such a significant association [15–17,19,20,22,23]. The potential reasons for the inconsistency of the results are still unknown. Therefore, in the present study, we performed a meta-analysis to systematically evaluate the potential association between prediabetes and the incidence of major adverse cardiovascular events (MACEs) in CAD patients after PCI. Specifically, the potential influences of study and patient characteristics on this association are explored by subgroup analyses.

## Methods

The present study was performed in accordance with the MOOSE (Meta-analysis of Observational Studies in Epidemiology) [24] and Cochrane’s Handbook [25] guidelines.

### Database search

We searched the databases of PubMed and Embase for relevant records, using the terms of “prediabetes” OR “pre-diabetes” OR “prediabetic state” OR “impaired fasting glucose” OR “impaired glucose tolerance”, combined with “percutaneous coronary intervention” OR “stent” OR “angioplasty” OR “revascularization” OR “reperfusion”. We limited the search to human studies published in English. A manual analysis of the reference lists of original and review articles was performed as a supplementation. The final search was performed on June 28, 2019.

### Inclusion and exclusion criteria

Studies were included if they met the following criteria: (1) full-length article in English; (2) designed as longitudinal follow-up studies; (3) including CAD patients that underwent PCI; (4) patients with prediabetes as exposure of interest at baseline; (5) documented the incidences of major adverse cardiovascular events (MACEs) a following PCI in patients with prediabetes and those with normoglycemia at admission; and (6) reported the multivariable adjusted risk ratios (RRs) and their corresponding 95% confidence intervals (CIs) for MACEs in patients with prediabetes compared to those with normoglycemia. The MACE was defined as a composite outcome of all-cause death, non-fatal myocardial infarction (MI), non-fatal stroke, repeated coronary revascularization and cardiac readmission. The diagnosis of prediabetes was based on the criteria of the original articles. For repeated reports of the same cohort, latest studies with the longest follow-up duration were included.

### Data extracting and quality evaluation

Database search, data extraction and quality assessment were independently performed by two authors, and discrepancies were resolved by consultation with the corresponding author. Data extracted include: (1) first author, location and design of the study; (2) number, mean age, diagnosis of the patients and types of PCI (primary or elective); (3) diagnostic criteria for prediabetes and number of patients with prediabetes; (4) follow-up durations and variables adjusted; and (5) outcome data for MACEs in CAD patients with prediabetes as presented in RRs and 95% CIs. Study quality evaluation was performed with the Newcastle–Ottawa Scale [26], which ranges from 1 to 9 stars and judges each study regarding three aspects: selection of the study groups; the comparability of the groups; and the ascertainment of the outcome of interest.

### Statistical analyses

Data of RRs and their corresponding stand errors (SEs) were calculated from 95% CIs or *P* values, and were logarithmically transformed to stabilize variance and normalized the distribution [25]. The Cochrane’s *Q* test and *I*^2^ test were performed to evaluate the heterogeneity among studies [27]. An *I*^2^ > 50% indicates significant heterogeneity. A random-effect model was applied since it incorporates the potential heterogeneity of the included studies and could lead to a more generalized result. Sensitivity analyses by removing individual study one at a time were performed to evaluate the stability of the results [28]. Subgroup analyses were performed to evaluate the impacts of study characteristics (including study design, sample size, CAD subtype, PCI type, definition of diabetes, follow-up duration, and adjustment of coronary artery severity) on the outcome. Potential publication bias was assessed by funnel plots with the Egger regression asymmetry test [29]. RevMan (Version 5.1; Cochrane Collaboration, Oxford, U.K.) and STATA software (Version 12.0; Stata Corporation, College Station, TX) were used for the statistical analyses.

## Results

### Results of literature search

The processes of database search and study identification were presented in Figure 1. Briefly, 587 studies were obtained via initial literature search, and 559 were excluded based on title and abstract because they were irrelevant to the study purpose. The remaining 28 studies underwent full-text review. Of them, sixteen were further excluded because one of them was not a follow-up study, six did not include patients that underwent PCI, four did not report MACE outcome, four were without available outcome data, and the other one did not include controls with normoglycemia. Finally, twelve follow-up studies were included [12–23].

**Figure 1:** Flowchart of database search and study identification

### Study characteristics and quality evaluation

The characteristics of the included studies are presented in Table 1. Overall, our meta-analysis included 10,048 CAD patients that underwent PCI from 12 follow-up studies [12–23]. These studies were designed as prospective cohort [12,15,16,18], retrospective cohort [13,14,17,18,20] or post-hoc analyses of the randomized controlled trials (RCTs) [21–23]. Two studies included patients with stable CAD [12,17], five studies included only patients with ST-segment elevation myocardial infarction (STEMI) [13,14,16,18,19], one with acute coronary syndrome (ACS) [23], while the other included a broad patients with CAD [20–22]. Primary PCI was applied in five studies [13,14,16,18,19], and elective PCI was applied in four studies [12,15,17,20]. A total of 3368 patients were with prediabetes at admission, as defined by the criteria with IFG and/or IGT in seven studies [12–17,22], with HbA1c in three studies [18–20], and IFG and/or HbA1c in two studies [21,23]. The mean age of the included CAD patients varied from 57.2 to 67.8 years, with proportions of male patients ranging from 66.5 to 85.8%. The follow-up durations varied from one to 52 months. Demographic factors, CAD risk factors, baseline cardiac function, coronary severity and medications for CAD were adjusted to a variable extent when presenting the RR and 95% CI for the association between prediabetes and MACEs. The Newcastle–Ottawa scale varied from 7 to 9 stars for the included studies.

**Table 1:** Characteristics of the included studies

Study	Design	Country	Patients	Sample size	PCI type	No. of prediabetic patients	Mean age	Male	Definitions of prediabetes	Follow-up duration	Variables adjusted	NOS
							Years	%		Months		
Dibra 2005	PC	German	Stable CAD	990	Elective	189	65.4	79.7	IFG (>100 mg/dl)	12	Age, gender, smoking, HTN, HC, previous MI, BMI, multivessel CAD, LVEF, SCr, using of β-blocker, ACEI/ARB and statins	9
Porter 2008	RC	Israel	STEMI	531	Primary	134	59.8	85.8	IFG (> 110 mg/dl)	1	Age, Killip Class, LVEF, renal function, anemia and three-vessel CAD	7
Fefer 2008	RC	Israel	STEMI	376	Primary	112	57.2	85.1	IFG (>100 mg/dl)	30	Age, gender, Killip Class I, previous MI, number of diseased vessels, LVEF and HTN	8
de la Hera 2009	PC	Spain	CAD excluding STEMI	338	Elective	121	66.5	80.1	IFG (> 110 mg/dl) or IGT	12	Age, indication of PCI, three-vessel or LM-CAD, LVEF, treatment with drug-eluting stents, IIb/IIIa inhibitors and statins	8
Knudsen 2011	PC	Norway	STEMI	224	Primary	105	57.4	83.1	IFG (> 110 mg/dl) or IGT	33	Age, gender, HTN, previous MI, smoking, BMI, elevated TG and TC, TnT and infarct size expressed as percent of ventricular mass	9
Kuramitsu 2013	RC	Japan	Stable CAD	376	Elective	236	67.8	82.2	IGT	52	Age, gender, TC, LDL-C and previous stroke	7
Shin 2016	RC	Korea	STEMI	2470	Primary	1475	62.1	77.4	HbA1c > 5.7%	12	Age, gender, BMI, LVEF, Killip class III or IV, troponin I and TC	7
Samir 2016	PC	Egypt	STEMI	208	Primary	96	74.8	72.7	HbA1c > 5.7%	6	Age, gender, BMI, smoking, HTN, LVEF, Killip class, troponin I, and TC and coronary lesion features	8
Kok 2018	RCT post-hoc	the Netherlands	Broad CAD patients including STEMI	2326	Both	324	64.1	71.8	IFG (>110 mg/dl) or HbA1c > 6.0%	12	Age, gender, smoking, HTN, HC, faimily history of CAD, previous MI, BMI and multivessel CAD	7
von Birgelen 2018	RCT post-hoc	the Netherlands	Broad CAD patients including STEMI	988	Both	132	61.9	78.2	IGT	12	Age, gender, HC, previous MI and previous revascularization	7
Choi 2018	RC	Korea	CAD excluding STEMI	674	Elective	242	62.3	66.5	HbA1c > 5.7%	24	Age, gender, smoking, HTN, HC, previous MI, BMI, multivessel CAD and LVEF	8
Farhan 2019	RCT post-hoc	US	ACS	547	Both	202	58.5	76.4	IFG (>110 mg/dl) or HbA1c > 5.7%	36	Age, gender, presence of thin-cap fibroatheroma, presence of minimal luminal area <4 mm^2^ and prior PCI	7

PC, prospective cohort; RC, retrospective cohort; RCT, randomized controlled trial; CAD, coronary artery disease; STEMI, ST-segment elevation myocardial infarction; ACS, acute coronary syndrome; IFG, impaired fasting glucose; IGT, impaired glucose tolerance; HbA1c, glycosylated hemoglobin; HTN, hypertension; HC, hypercholesterolemia; MI, myocardial infarction; BMI, body mass index; LVEF, left ventricular ejection fraction; SCr, serum creatinine; ACEI, angiotensin converting enzyme inhibitor; ARB, angiotensin II receptor blocker; LM, left main; TC, total cholesterol; TG, triglyceride; TnT, troponin T; TnI, troponin I; LDL-C, low density lipoprotein cholesterol; PCI, percutaneous coronary intervention; NOS, the Newcastle–Ottawa Scale;

### Association between prediabetes and MACEs following PCI

Moderate heterogeneity was detected for the included follow-up studies (*P* for Cochrane’s *Q* test = 0.08, *I*^2^ = 39%). Pooled results with a random-effect model showed that patients with prediabetes at admission were with significantly higher risk of MACEs during follow-up after PCI compared to those without normoglycemia (adjusted RR: 1.53, 95% CI: 1.25–1.87, *P* < 0.001; Figure 2). Sensitivity analyses by excluding one study at a time did not change the results (RR: 1.45–1.66, *P* all < 0.05). Subgroup analyses indicated that the association between prediabetes and higher risk of MACEs remained significant regardless of the study design, sample size, CAD subtype, PCI type, definition of diabetes or follow-up duration (Table 2). Moreover, patients with prediabetes had higher significantly risk of MACEs in studies with adjustment of coronary lesion severity (RR: 1.79, 95% CI: 1.46–2.19, *P* < 0.001), but the association became insignificant in studies without adjustment of the coronary lesion severity (RR: 1.23, 95% CI: 0.97–1.55, *P* = 0.09).

**Figure 2:** Forest plots for the meta-analysis of the incidence of MACE in patients with prediabetes compared to those with normoglycemia after PCI

**Table 2:** Subgroup analyses

Study characteristics	Datasets number	RR (95% CI)	*I*^2^	*P* for subgroup effect	*P* for subgroup difference
**Study design**					
PC	4	1.51 [1.13, 2.02]	63%	0.005	
RC	5	1.42 [1.14, 1.77]	44%	0.002	
Post-hoc analysis of RCT	3	1.77 [1.30, 2.42]	0%	< 0.001	0.51
**Sample size**					
<500	5	1.48 [1.15, 1.91]	46%	0.002	
≥ 500	7	1.55 [1.28, 1.87]	43%	< 0.001	0.79
**CAD subtype**					
STEMI only	5	1.40 [1.12, 1.75]	52%	0.003	
Others	7	1.64 [1.33, 2.02]	31%	< 0.001	0.32
**PCI type**					
Primary	5	1.40 [1.12, 1.75]	52%	0.003	
Elective	4	1.53 [1.16, 2.03]	55%	0.003	
Both	3	1.77 [1.30, 2.42]	0%	< 0.001	0.48
**Definition of prediabetes**					
FPG and/or IGT	7	1.59 [1.27, 1.98]	34%	< 0.001	
HbA1c	3	1.31 [1.01, 1.72]	63%	0.04	
IFG or HbA1c	2	1.75 [1.26, 2.44]	32%	< 0.001	0.37
**Follow-up duration (months)**					
≤12	7	1.53 [1.26, 1.86]	61%	< 0.001	
>12	5	1.51 [1.19, 1.94]	0%	< 0.001	0.95
**Adjustment of coronary severity**					
Yes	7	1.79 [1.46, 2.19]	29%	< 0.001	
No	5	1.23 [0.97, 1.55]	0%	0.09	0.03

PC, prospective cohort; RC, retrospective cohort; RCT, randomized controlled trial; CAD, coronary artery disease; STEMI, ST-segment elevation myocardial infarction; HbA1c, glycosylated hemoglobin.

### Publication bias

The funnel plots for the meta-analysis of the association between prediabetes and risk of MACEs are shown in Figure 3. The funnel plots were symmetry on visual inspection. Egger’s regression test also indicated low risk of publication bias (*P* = 0.426).

**Figure 3:** Funnel plots for the meta-analysis

## Discussion

In this meta-analysis of longitudinal follow-up studies, we found that compared to patients with normoglycemia, CAD patients with prediabetes at admission have significantly higher risk of MACEs after PCI. Further subgroup analyses indicated that the potential predictive role of prediabetes for these patients is consistent regardless of the study characteristics of study design, sample size, CAD subtype, PCI type, definition of diabetes or follow-up duration, and even after adjustment of the severity of coronary lesions. Taken together, these results demonstrated that prediabetes at admission may be an independent predictor of poor prognosis after PCI in CAD patients without DM.

To the best of our knowledge, our study is the first meta-analysis that evaluated the potential prognostic role of prediabetes at admission for CAD patients that underwent PCI. We found that prediabetes at admission is independently associated with higher risk of MACEs in CAD patients after PCI, which has the following clinical implications. First, prevalence of prediabetes is high in CAD patients. The pooled prevalence of prediabetes in our included CAD patients for PCI is 33.5%, which is similar to the previous reports [30–32]. Second, compared those with normoglycemia at admission, patients with prediabetes have poor prognosis after PCI. Since the robustness of the results was validated by sensitivity analyses and subgroup analyses according to multiple study characteristics, our study strongly demonstrated that prediabetes is an independent prognostic factor for patients after PCI. These findings support the screening for abnormal glycemic metabolism in CAD patients that underwent PCI. Moreover, in view of the high prevalence of prediabetes in CAD patients, these findings highlight the importance to validate the hypothesis that whether interventions targeting prediabetes could improve the prognosis in these patients.

The potential pathophysiological mechanism underlying the independent association between prediabetes and incidence of MACEs after PCI remains to be determined. Currently, we could not exclude the chance that the potential association between prediabetes and poor prognosis after PCI is mainly driven by the progression of prediabetes to DM in substantial patients [33]. However, it has been confirmed by previous studies that patients with prediabetes may already have early but severe coronary lesions. Indeed, an early intravascular ultrasound (IVUS) study showed that patients with IGT were more likely to have lipid-rich coronary plaque as compared with patients with normoglycemia, which may be mediated by insulin resistance [34]. Furthermore, it has been suggested that patients with prediabetes had a smaller coronary size and diffuse coronary narrowing compared to those with normoglycemia, which may cause increased risk for MACEs after PCI [35]. Restenosis has been confirmed as a major determinant of MACEs after revascularization [36]. Accumulating evidence from epidemiological studies and experimental studies has shown that overactivated systematic inflammation plays an important role in the pathogenesis of restenosis [37,38]. Interestingly, patients with prediabetes have been associated with insulin resistance and activated inflammatory response, which therefore may be vulnerable to restenosis after revascularization. In a mouse model of wire injury induced femoral artery neointimal formation, maintaining of insulin sensitivity is associated with decreased level of neointimal growth [39]. In a study of 136 patients that underwent elective percutaneous coronary intervention with the second generation drug-eluting stents, insulin resistance has been related with the severity of intra-stent neointimal tissue proliferation [40]. These findings implied a potential association between prediabetes, insulin resistance, inflammation and restenosis after revascularization. Further studies are needed to evaluate the potential pathophysiological mechanisms underlying the prognostic role of prediabetes in patients after PCI.

Our study also highlighted the importance of applying novel therapeutic approaches to reduce the risk of MACEs in patients with glycemic dysregulation, including prediabetes. First, identification of novel key molecular and signaling pathway in restenosis is fundamental to develop target therapeutic strategies against the risk of MACEs after PCI. Recently, inhibition of p110δ isoform of phosphoinositide 3-kinase (PI3K) has been shown to prevent inflammatory response and restenosis after artery injury [41], demonstrating a potential therapeutic direction via targeted manner such as gene therapy [42]. In addition, some novel techniques and instruments may bring more favorable outcomes in patients underwent percutaneous interventional therapy, such as provisional stenting for the obstructive lesions of the popliteal artery [43], using of newer-generation stents in PCI (including the everolimus-eluting stent [44], and the polymer-free sirolimus- and probucol-eluting stent [45].). Interestingly, a previous study showed that everolimus-eluting stents compared with paclitaxel-eluting stents resulted in substantial 2-year reductions in MACE risks in non-diabetic patients, but not in diabetic patients [46]. It has not been determined whether the superiority of everolimus-eluting stent remains in patients with prediabetes. Future studies are needed in this era.

The strengths of our study include the overall large sample size of the included patients and the robustness of the findings as evaluated by sensitivity and subgroup analyses. Moreover, our study also has some limitations. First, we performed subgroup analyses to confirm that the association between prediabetes and risk of MACEs after PCI are consistent in studies with prediabetes defined by IFG/IGT, HbA1c and IFG/HbA1c. However, the definitions of prediabetes varied within the included studies and the limited number of available studies prevented further analyses to determine the optimal definition of prediabetes that confers the highest risk for MACEs as compared to patients with normoglycemia. Further studies are needed to determine the optimal definition for prediabetes regarding their association with adverse events after PCI. Second, as a meta-analysis of observational studies, although we combined the most adequately adjusted RR, we could not exclude the residual factors that may confound the association between prediabetes and risk of MACEs after PCI. In addition, a causative relationship between prediabetes and increased risk of MACEs after PCI could not be indicated based on our meta-analysis. In the future, RCTs evaluating the impact of interventions targeting glucose metabolism on clinical outcomes in patients with prediabetes after PCI are needed. Currently, lifestyle modifications are generally recommended for people with prediabetes. However, whether lifestyle modifications are adequate for improve the prognosis in high-risk patients with prediabetes, such as those after PCI, deserves further investigation.

In conclusion, prediabetes at admission may be an independent predictor of higher incidence of MACEs after PCI in CAD patients without DM. These findings support the screening of abnormal glycemic metabolism in patients receiving PCI. The potential benefits of interventions targeting abnormal glycemic metabolism clinical outcomes in patients with prediabetes after PCI should be evaluated in the future.

## Abbreviations

CAD: coronary artery disease
IFG: impaired fasting glucose
IGT: impaired glucose tolerance (IGT)
MACE: percutaneous coronary intervention
PCI: major adverse cardiovascular event
